# Role of Gas6 and TAM Receptors in the Identification of Cardiopulmonary Involvement in Systemic Sclerosis and Scleroderma Spectrum Disorders

**DOI:** 10.1155/2020/2696173

**Published:** 2020-05-12

**Authors:** Mattia Bellan, Arnaldo Dimagli, Cristina Piccinino, Ailia Giubertoni, Aurora Ianniello, Federico Grimoldi, Maurizio Sguazzotti, Alessandra Nerviani, Michela Barini, Alessandro Carriero, Carlo Smirne, Michela Emma Burlone, Cristina Rigamonti, Rosalba Minisini, Livia Salmi, Matteo Nazzareno Barbaglia, Luigi Mario Castello, Daniele Sola, Paolo Marino, Gian Carlo Avanzi, Mario Pirisi, Pier Paolo Sainaghi

**Affiliations:** ^1^Department of Translational Medicine, Università del Piemonte Orientale, UPO, Novara, Italy; ^2^Internal Medicine Division, Immunorheumatology Unit, CAAD (Center for Autoimmune and Allergic Diseases), “Maggiore della Carità” Hospital, Novara, Italy; ^3^IRCAD, Interdisciplinary Research Center of Autoimmune Diseases, Novara, Italy; ^4^Division of Cardiology, “Maggiore della Carità” Hospital, Corso Mazzini 18, 28100 Novara, Italy; ^5^Rheumatology Outpatient Unit, ASL Novara, Italy; ^6^Barts and The London School of Medicine and Dentistry, William Harvey Research Institute, Queen Mary University of London, London, UK; ^7^Division of Radiology, “Maggiore della Carità” Hospital, Novara, Italy

## Abstract

**Background:**

Few biomarkers are available for early identification of pulmonary arterial hypertension (PAH) and interstitial lung disease (ILD) in systemic sclerosis (SS) and scleroderma spectrum disorders (SSD).

**Aims:**

To evaluate Gas6, sAxl, and sMer as biomarkers for cardiopulmonary complications of SS and SSD.

**Methods:**

In a cross-sectional observational study, we recruited 125 consecutive patients, affected by SS and SSD and referred to a tertiary-level pulmonary hypertension outpatient clinic. All patients underwent a comprehensive evaluation for identification of PAH and ILD. Gas6, sMer, and sAxl concentrations were measured with ELISA protocols, and concentrations were compared according to PAH or ILD.

**Results:**

Nineteen subjects had pulmonary hypertension (PH) (14 PAH), and 39 had ILD (6 severe). Plasma sMer was increased in PAH (18.6 ng/ml IQR [11.7-20.3]) with respect to the absence (12.4 [8.0-15.8]) or other form of pulmonary hypertension (9.6 [7.4-12.5]; K–W variance *p* < 0.04). Conversely, Gas6 and sAxl levels were slightly increased in mild ILD (25.8 ng/ml [19.5-32.1] and 24.6 [20.1-32.5]) and reduced in severe ILD (16.6 [15.0-22.1] and 15.5 [14.9-22.4]) in comparison to no evidence of ILD (23.4 [18.8-28.1] and 21.6 [18.1-28.4]; K–W, *p* ≤ 0.05). Plasma sMer ≥ 19 ng/ml has 50% sensitivity and 92% specificity in PAH identification (area under the ROC curve (AUC) 0.697, *p* < 0.03). Values of Gas6 ≤ 24.5 ng/ml and of sAxl ≤ 15.5 ng/ml have 100% and 67% sensitivity and 47% and 86% specificity, respectively, in identifying severe ILD (Gas6 AUC 0.787, *p* < 0.001; sAxl AUC 0.705, *p* < 0.05).

**Conclusions:**

The assay of Gas6 sAxl and sMer may be useful to help in the identification of PAH and ILD in SS and SSD patients. The Gas6/TAM system seems to be relevant in cardiopulmonary complications of SS and SSD and merits further investigations.

## 1. Introduction

Pulmonary arterial hypertension (PAH) and interstitial lung disease (ILD) are severe and potentially life-threatening complications of systemic sclerosis (SS) and scleroderma spectrum disorders (SSD), as mixed connective tissue diseases (MCTD) and SS overlap with other connective tissue diseases (CTDs) [1].

PAH is defined by the presence of a mean pulmonary arterial pressure (mPAP) equal to or greater than 25 mmHg and a pulmonary capillary wedge pressure (PCWP) equal to or less than 15 mmHg, assessed during invasive right heart catheterization (RHC) at rest [2]. PAH associated with CTD (CTD-PAH) has been reported from 20% to 30% in SS and SSD [3], and its prognosis is even poorer than that of the idiopathic form of PAH (IPAH) [4]. Indeed, an early diagnosis and a well-timed treatment are able to improve the prognosis in this setting [5]. Currently, the two-step algorithm (DETECT) is the most widely used screening tool for SS patients [6], but the search for novel biomarkers with diagnostic and prognostic significance is still warranted.

Connective tissue disease associated with interstitial lung diseases (CTD-ILD) are a heterogeneous group of conditions characterized by chronic inflammation and/or parenchymal fibrosis within the contest of CTD [7, 8]. The complex diagnostic approach and the faintness of diagnostic criteria make the estimation of CTD-ILD prevalence very difficult, ranging from 15% to 90% according to different series [9–11]. The presence of a severe ILD is one of the most prominent negative prognostic factor in the clinical course of a CTD, being the most frequent cause of death in SS [12]. As for PAH, the early detection of lung involvement and the stratification of the risk of fibrosis progression are quintessential for modifying prognosis with early, appropriate treatment.

Growth arrest specific 6 (Gas6) is a vitamin K-dependent protein, identified as ligand for a tyrosine-kinase receptors family, collectively named TAM (acronym of Tyro3, Axl, and Mer) [13]. TAM receptors are variably expressed in many tissues and can be found as a soluble form in the bloodstream (sTyro3, sAxl, and sMer, respectively) [14]. These soluble forms are the result of the proteolytic cleavage by two metalloproteinases, ADAMTS 17 and ADMATS 10, and probably act as decoy receptors for the ligands [13, 15]. The Gas6/TAM system is highly pleiotropic and involved in several functions: among them, it seems to have a relevant role in the regulation of inflammatory response [16, 17], tissue repair and fibrosis development [14], and vascular integrity [18, 19]. Consistently, an impairment of the Gas6/TAM system has been associated with the development of autoimmune diseases, as demonstrated by the murine model of triple knock-out for the TAM receptors [20].

On these bases, Gas6 and its soluble receptors have been proposed as biomarkers in different human conditions [21, 22], specifically in autoimmune diseases [23–26]. In the present study, we aim to evaluate Gas6 and sAxl and sMer as potential biomarkers for cardiopulmonary complications of SS and SSD.

## 2. Materials and Methods

### 2.1. Patients

We performed a cross-sectional observational study. From October 1, 2016, to April 20, 2018, we recruited one hundred and twenty-five consecutive patients, affected by SS and SSD and referred to the Pulmonary Hypertension Outpatient Clinic of the Cardiology Department, A.O.U. “Maggiore della Carità”, Novara, Italy.

The study protocol was approved by the institutional ethical committee and conducted in strict accordance with the principles of the Declaration of Helsinki. Written informed consent was obtained from all individual participants included in the study.

We included all the consecutive patients willing to participate, with one of the following diagnoses:

- SS according to 2013 ACR/Eular classification criteria [27], including overlap with other rheumatic diseases
- MCTD according to Kasukawa criteria [28]

We applied the following exclusion criteria:

- Age < 18 years
- Impossibility to undergo the required cardiopulmonary assessment

The design of the present cross-sectional observational study and part of the methods were already been described elsewhere [29].

### 2.2. Procedures

All patients underwent a comprehensive medical history, including the assessment of cardiovascular risk factors, comorbidities, rheumatologic disease, and drug history. A physical examination was performed by an experienced clinician; anthropometric data were recorded.

The patients underwent an appropriate biochemistry panel. The serological profile of autoantibodies was recorded.

The assessment of each patient consisted of

- 12-lead electrocardiogram with 6-limb and 6 precordial leads with paper speed set at the standard rate of 25 mm/s
- Posteroanterior and lateral chest X rays
- Pulmonary function tests (PFTs): the test was performed using a standardized equipment and technique with a spirometer. The device was connected to a computer employing the software “Medisoft Expair 1.28.20”. The following standardized measurements were evaluated: forced vital capacity (FVC), forced expiratory volume in one second (FEV1), and FEV1/FVC% (also known as the Tiffeneau index). We also evaluated the diffusing capacity of the lung for carbon monoxide (DLCO), measured with the single-breath Jones-Meade protocol. Once the mouthpiece and the nose clip were in place, the subject made a maximal expiration and then, with a maximal inspiration inhaled a gas blend containing carbon monoxide (0.3%) and other inert gases (0.3% CH4). Then, the patient was asked to hold his/her breath for about 10 seconds and exhale afterward. During the expiration, alveolar air was analyzed: the ratio between carbon monoxide in inspired gas and carbon monoxide in exhalated air determined the diffusion of carbon monoxide. Predicted DLCO was corrected for hemoglobin, and alveolar volume was assessed
- Transthoracic echocardiography (TTE) was performed using the Vivid 7 or E9 cardiovascular ultrasound machine by GE Medical Systems (Horten, Norway) with a 1.7/3.4 MHz tissue harmonic transducer. All data were obtained in standardized patient positions, according to the standards of the American Society of Echocardiography. The test was performed by an expert, pulmonary hypertension echocardiographer. The following parameters were generated [30]: systolic pulmonary pressure (sPAP), right atrium area (RAA), right ventricle diameter (RVD), and ejection fraction (EF). Right ventricle systolic function was evaluated by estimating the tricuspid annular plane systolic excursion (TAPSE).

According to the application of international guidelines [2], those patients with a suspected PAH underwent right heart catherization (RHC, *n* = 15). PAH was defined by mean pulmonary artery pressure (mPAP) ≥ 25 mmHg, pulmonary capillary wedge pressure ≤ 15 mmHg, and pulmonary vascular resistance > 3 wood units. Whenever contraindications to RHC occurred, pulmonary hypertension was diagnosed based on echocardiography-estimated sPAP ≥ 35 mmHg and additional high probability criteria, according to 2015 ESC/ESR guidelines. [2].

Those patients with a clinical and instrumental suspicion of CTD-ILD underwent a high-resolution computed tomography (HRCT) (*N* = 58) assessed by an expert, ILD radiologist. ILD was defined by the presence of ground glass opacities (GGO) and/or reticular pattern. Moreover, the extension of pulmonary fibrosis was measured with the Goh score [31] and a modified Kazerooni score [32]. When applying the Goh score, five thin-section CT slices were considered (level of origin of great vessels, tracheal carina, superior pulmonary veins, immediately above the right hemidiaphragm, and one halfway between the third and the fifth slices) and for each one, a quantitative assessment of fibrosis was performed. A mean value from the five sections was obtained. Following these assessments, patients were divided into two categories: limited ILD (fibrosis less than 10% or ranging from 10% to 30% with an FVC greater than 70%) and severe ILD (fibrosis greater than 30% or ranging from 10% to 30% with an FVC less than 70%) [31].

The *modified* Kazerooni score semiquantitatively evaluated the severity of fibrosis in each out of five slices, instead of three as described in the original paper, as follows: (0) no fibrosis, (1) fibrosis ≤ 5%, (2) fibrosis < 25%, (3) fibrosis from 25% to 49%, (4) fibrosis from 50% to 75%, and (5) fibrosis > 75% [32].

Gas6, sMer, and sAxl plasmatic concentrations were measured. Blood sample was drawn from each patient and collected in a 4 ml Vacutainer lavender K2-EDTA tube. Within an hour, the blood sample was centrifuged and then stored at -80°C.

Plasma sAxl concentration was measured using the DuoSet® ELISA R&D Systems DY154 commercial kit, according to the manufacturer's protocol. The aliquots were diluted 1 : 75 in PBS and bovine serum albumin 1% (reagent diluent). The dilution factor was chosen according to the previous experience of our laboratory.

Plasma sMer concentration was measured using the DuoSet® ELISA R&D Systems DY6488 commercial kit, according to the manufacturer's protocol. The samples were diluted 1 : 5 in reagent diluent, according to previous analysis in our laboratory.

Plasma Gas6 concentration was measured according to the protocol described by Alciato et al. for plasma [33] and other body fluids [34]. A 96-well plate (NUNC Products, Thermo Scientific Inc. MA, USA) was coated with the primary antibody, Goat-IgG anti-human Gas6 (R&D Systems, Minneapolis, USA), and left incubated overnight at room temperature. The antigen was detected using a Goat-IgG biotinylated anti-human Gas6 antibody (R&D Systems, Minneapolis, USA), streptavidin conjugated with horseradish peroxidase (Sigma, St. Louis, MO, USA), and the chromogen tetramethylbenzidine (Sigma, St. Louis, MO, USA). The reaction was blocked with sulfuric acid 2N, and absorbance detected at 450 with a reference wavelength set at 570 nm. Optical density was fitted versus nominal concentration by applying a four-parameter logistic regression to the calibration curve prepared in BSA (bovine serum albumin, further purified fraction V, ≥98%, Sigma, St. Louis, MO, USA).

### 2.3. Statistical Analysis

Anthropometric, clinical, and biochemical data were recorded in a database and analyzed by the statistical software package MedCalc v.18.10.2 (MedCalc Software, Broekstraat 52, 9030, Mariakerke, Belgium). The normality of Gas6, sMer, and sAxl distribution was assessed by the Shapiro-Wilk test; following the nonnormal distribution observed, we performed a nonparametrical analysis.

The measures of centrality and dispersion of data chosen were medians and interquartile range (IQR). Medians were compared between groups by the Mann–Whitney and Kruskal–Wallis (K–W) and post hoc tests. Correlations between continuous variables were performed by Spearman's rank test. To test the diagnostic performance of the studied biomarkers, receiver operating characteristics curves were built, with calculation of the respective areas under the curve (AUC). The level of significance chosen for all statistical analysis was 0.05 (two-tailed).

## 3. Results

Table 1 reports general features of the 125 patients enrolled; among patients affected by SS or SS overlap, 78% showed a limited cutaneous involvement. After evaluation of cardiopulmonary workup, 19 (15%) subjects received a diagnosis of PH, of whom 14 CTD-PAH, 2 PH due to the left heart, and 3 due to lung disease. Additionally, 39 (31%) patients were affected by ILD, which was characterized by a severe functional impairment in 6 (5%) of them.

Gas6, sAxl, and sMer median plasma levels were not different according to the extent of cutaneous involvement (limited vs diffuse), sex, disease duration (<5 vs ≥5 years), smoking status, liver disease, and immunosuppressive and vasodilator treatments (*p* = NS).

We compared the median values of Gas6, sAxl, and sMer according to the presence of pulmonary hypertension. Data are reported in Table 2. As evident, sMer plasma levels are increased in CTD-PAH, while Gas6 and sAxl were similar among groups. No significant correlation was observed between sMer and PAP either assessed by echocardiography or by RHC (*p* = NS).

With respect to biomarker variations according to the presence of CTD-ILD, we observed a trend towards a slight increase of Gas6 and sAxl in mild ILD. Conversely, we observed a more evident reduction for both in severe ILD. sMer concentrations were similar among groups (also see Table 2). Notably, Gas6 and sAxl were related to the extent of ILD at CT scan measured with the *modified* Kazerooni score; in fact, a significant negative correlation with the extent of fibrosis is evident both for Gas6 (*r*: -0.46, *p* < 0.03) and sAxl (r: -0.45, *p* < 0.03).

We finally evaluated the diagnostic accuracy of sMer in diagnosing PAH; a sMer threshold > 19 ng/ml has a 50% sensitivity and a 92% specificity in diagnosing PAH (Figure 1(a)) with a positive predictive value (PPV) of 44% and a negative predictive value (NPV) of 94%. Moreover, we evaluated Gas6 and sAxl diagnostic accuracy in the identification of ILD; a Gas6 threshold ≤ 24.5 ng/ml has a 100% sensitivity, 47% specificity, 46% PPV, and 100% NPV; sAxl < 15.5 ng/ml is 67% sensitive and 86% specific in identifying severe ILD in our population (Figures 1(b) and 1(c)) with 67% and 85% PPV and NPV, respectively.

## 4. Discussion

Patients affected by SS and/or SSD have a reduced life expectancy than age- and sex-related population; this is mainly determined by two severe cardiopulmonary complications, CTD-PAH and CTD-ILD [12]. Since a timely diagnosis is a sdeterminant to implement appropriate treatments to obtain better outcomes [5], a combination of biomarkers is warranted to increase the ability to screen patients at risk in addition to current methods.

We designed the present study to investigate the role of the measurement of Gas6 protein and of the soluble forms of its receptors Axl and Mer in plasma of patients with SS and SSD to identify either CTD-PAH or CTD-ILD; our data support the assay of sMer as biomarker of PAH in CTD patients. Conversely, Gas6 and sAxl determination might contribute to the identification of CTD-ILD. These results need to be discussed looking at the current literature evidences.

In our population, sMER concentration in plasma was increased in CTD-PAH, while neither that of Gas6 nor of sAxl was different according to this complication. Endothelial dysfunction is known to be a key impairment of CTD-PAH sustained by a mismatch of mediators acting as vasodilators in favour of vasoconstrictors; this process evolves with the activation of vascular remodelling towards an increase of vascular tone mediated by the endothelium and vascular smooth muscle cell (VSMC) activation [35]. Gas6/TAM interplay is known to be involved in vessel wall homeostasis: Gas6 was isolated from aortic endothelial cells, and it has a trophic effect on vessel walls; additionally, the Gas6/TAM system is activated in case of vessel damage or in human atherosclerotic plaque formation [14, 36]. Possibly, sMER increase in these patients could be an expression of endothelial stress and dysfunction, typical of PAH. One additional possible explanation comes from the other mainstay of the pathogenesis of CTD-PAH, the presence of persistent inflammation of pulmonary vessel walls [35]. TAM receptors, indeed, are involved in regulation of innate immunity, being upregulated in activated antigen-presenting cells (APCs) through type I interferon (IFN) signalling that determines the activation of suppressor of cytokine signalling proteins (SOCS1 and SOCS3) which, in turn, dampens the inflammatory response [37, 38]. Additionally, Gas6, through TAM receptors, limits proinflammatory cytokine production of APCs, through the inhibition of toll-like receptor (TLR) downstream signal [17]. In particular, Mer seems to be more relevant than Axl in apoptotic bodies' recognition favouring phagocytosis/efferocytosis and in the reduction of proinflammatory cytokine production in vitro and in vivo models [39, 40]. Therefore, the elevation of sMer in these patients may be the combination of a dysfunction of the endothelium and VSMCs and of an impairment of mechanisms that dampen inflammation of the pulmonary artery vessel wall. Since soluble TAM receptors seem to act as decoy receptors [15, 41], an increment of sMer can be considered an indirect evidence of an impairment of Mer receptorial function. In any case, this pathophysiological discussion is merely speculative and merits an ad hoc investigation.

In the population studied, both Gas6 and sAxl plasma values were significantly reduced in patients with severe ILD; additionally, a mild increment is observed in milder forms; in contrast to patients with CTD-PAH, sMer is not changed. There are several evidences of the role of the Gas6/Axl system in the modulation of fibrotic evolution of tissues affected by chronic inflammation; in particular, Gas6 is relevant in the modulation of inflammation and fibrosis of the liver and it marks the evolution to cirrhosis [42]. Gas6^−/−^ mice shows an increased damage of the liver and an impairment in healing after carbon tetrachloride administration; rGas6 administration limits this damage but in turn favours fibrotic repair [43–45]. Consistently, Gas6 enhances survival of hepatic stellate cells (HSCs) and of HSCs activated into myofibroblastic cells (HSCs/MFBs) which are involved in the production of cytokines and matrix protein during liver injury [46]. The relevance of the Gas6/Axl axis in liver fibrosis has also been described in humans. In fact, plasma Gas6 concentrations are increased in hepatic cirrhosis and correlate with disease evolution [47] and with liver elastography measures, helping to identify severe complications as oesophageal varices [48, 49]. Accordingly, the slight increase of plasma Gas6 and sAxl in mild CTD-ILD can be the expression of evolution of chronic inflammation into interstitial fibrosis in the lung, either as a marker of the fibrosis progression or as the indicator of an impairment of the Gas6/Axl system in the control of inflammation; this interpretation is in line with recent reports where Gas6 was observed to increase peribronchial fibrosis in allergic airway disease [50, 51]. Additionally, Gas6 and Axl expressions were observed to increase in lung tissues and fibroblasts obtained from patients affected by idiopathic pulmonary fibrosis, a severe chronic fibrotic disease of the lung which shares several clinical and pathophysiological features with CTD-ILD [52]. Our finding of a reduction of Gas6 and sAxl in patients with severe ILD is only in apparent contrast with this explanation. In fact, on one hand, it may derive from a reduction of the lung tissue due to severe fibrosis or to the fact that in advanced ILD, the fibrotic evolution becomes independent from the initial chronic inflammation trigger. Anyway, also in this case, our pathophysiological discussion is merely speculative and merits further specific investigations.

### 4.1. Clinical Scenario

Moving to a more clinical point of view, the early detection of CTD-PAH is still a clinical challenge being this complication burdened with a high morbidity and mortality and an early diagnosis related to a better prognosis [1, 5]. The current screening strategy for PAH in these patients includes PFTs with DLCO, TTE and measurement of NT-proBNP, and the referral for RHC if positive results are obtained [53]. The recently proposed DETECT algorithm, which has been validated to stratify patients at risk to be referred to RHC, includes clinical, laboratory, and instrumental variables [6]. The two biomarkers included in the algorithm are NT-proBNP and urate are nonspecific for CTD-PAH [6]; in this contest, the measurement of sMER, which displayed a good diagnostic accuracy for PAH in SS and SSD patients, could be an additional tool to improve PAH detection algorithms.

Similarly, very few biomarkers have been proposed up till now for ILD detection in patients with SS, mainly proteins associated with damage and turnover of alveolar epithelial cells as lung epithelium-derived surfactant protein (SP-D), glycoprotein Krebs von den Lungen-6 (KL-6), CCL18, and soluble OX40 [54]. Recently, in a large cohort study of patients with SS, it was observed that SP-D was the most accurate for diagnosis, while KL-6 was related to severity of SSc-ILD; finally, CCL18 was the best prognostic factor for ILD progression [55]. It should be pointed out that both Gas6 and sAxl displayed a good accuracy in ILD identification in our cohort (AUC of 0.787 and 0.705, respectively) similar to that reported for KL-6 (0.689) [55]; if direct comparisons are inappropriate due to differences in study design, we can propose the sAxl/Gas6 assay as an additional tool for identification of ILD in patients affected by SS and SSD.

It is worth to be underlined that the Gas6/TAM system seems to be relevant for both complications of SS and SSD patients highlighting its possible pathogenetic role and utility in the diagnostic process.

### 4.2. Limitations

Some limitations of our study may interfere with the interpretations of the results: firstly, many patients were already receiving a treatment either for PAH or for CTD-ILD and this fact could have influenced the biomarker values measured in plasma; in second instance, the present study has a cross-sectional design that can limit interpretation of results in particular in terms of confounding factors, and a longitudinal cohort is needed for confirmation; our aim is to build a prospective cohort to evaluate Gas6/sAxl/sMer in comparison with other biomarkers at the development of CTD and PAH and during follow-up to establish a prognostic role. Additionally, a control group of healthy subjects would have been desirable; however, since our aim was not to evaluate the performance of such molecules in diagnosing SS and SSD but if these molecules are candidate biomarkers for cardiopulmonary complications, the importance of a control group may somewhat be lessened. In third instance, the number of cases of CTD and PAH was limited in number but in line to the expected prevalence. Finally, the lack of histopathological evaluations of analytes in pathological tissues further limits pathophysiological interpretations.

## 5. Conclusion

In conclusion, we have demonstrated that the assay of Gas6 and its receptors sAxl and sMer is a useful tool to help to establish if a patient affected by SS or SSD has developed either PAH or ILD; sMer displayed a good diagnostic accuracy for PAH while Gas6 and sAxl for ILD. Our results have also possible pathophysiological implications since the Gas6/TAM receptors system seems to be relevant in both PAH and ILD evolutions of SS and SSD patients and merits further investigations.

## Figures and Tables

**Figure 1:** (a) ROC curve for sMer in diagnosing PAH. Area under the ROC curve (AUC) 0.697, *p* < 0.03. (b) ROC curve for Gas6 in diagnosing severe ILD. AUC 0.787, *p* < 0.001. (c) ROC curve for sAxl in diagnosing severe ILD. AUC 0.705, *p* < 0.05.

**Table 1:** Characteristics and main comorbidities of the study population. The continuous variables are expressed as median (interquartile range), while the categorical variables as number (and frequency %).

Age, years	66 [56-75]
Gender, F/M	113/12
Disease duration, years	8 [3-13]
Smoking status, no/past smoker/active smoker	87(70)/20(16)/18(14)
Arterial hypertension	66 (57)
COPD	14 (11)
Cardiac disease^∗^	21 (17)
Liver disease/liver cirrhosis	18 (14)/0(0)
SS/MCTD/SS overlap	94(75)/13(10)/18(15)
Digital ulcer (past/active)	64(51)/13(10)
Anti-centromere/anti-Scl70/anti-U1RNP	67(54)/30(24)/28(22)
Arterial vasodilators: ERA/PDE5-I/iloprost	18(14)/7(6)/60(48)
PDN/HCQ/MTX	44(35)/66(53)/12(9)

Abbreviations: F: female; M: male; COPD: chronic obstructive pulmonary disease; SS: systemic sclerosis; MCTD: mixed connective tissue disease; SSD: scleroderma spectrum disorder; PAH: pulmonary arterial hypertension; ERA: endothelin receptor antagonist; PDE5-I: phosphodiesterase 5 inhibitor; PDN: prednisone; HCQ: hydroxychloroquine; MTX: methotrexate. ^∗^Chronic heart failure and/or coronary artery disease.

**Table 2:** Comparison of Gas6, sAxl and sMer according to cardiopulmonary involvement.

	ILD			K–W	Post hoc
	No (*N* = 86)	Mild (*N* = 33)	Severe (*N* = 6)		
Gas6 (ng/ml)	23.4 [18.8-28.1]	25.8 [19.5-32.1]	16.6 [15.0-22.1]	6.12, *p* < 0.05	No vs mild *p* < 0.05 Mild vs severe *p* < 0.04
sAxl (ng/ml)	21.6 [18.1-28.4]	24.6 [20.1-32.5]	15.5 [14.9-22.4]	5.73, *p* = 0.05	n.s.
sMer (ng/ml)	12.9 [8.5-16.0]	12.3 [8.1-16.6]	7.4 [5.4-17.1]	n.s.	n.s.

	PH			K–W	Post hoc
	No (*N* = 106)	CTD-PAH (*N* = 14)	Other PH (*N* = 5)		
Gas6 (ng/ml)	23.3 [18.5-28.1]	24.9 [18.8-33.9]	23.5 [23.3-31.9]	n.s.	n.s.
sAxl (ng/ml)	22.1 [18.2-30.1]	24.8 [20.0-28.2]	21.1 [15.6-23.3]	n.s.	n.s.
sMer (ng/ml)	12.4 [8.0-15.8]	18.6 [11.7-20.3]	9.6 [7.4-12.5]	6.44, *p* < 0.04	No vs CTD-PAH *p* < 0.05

Abbreviations: ILD: interstitial lung disease; CTD-PAH: connective tissue disease-related pulmonary arterial hypertension; PH: pulmonary hypertension; K–W, Kruskal–Wallis analysis of variance.

## Data Availability

Data are available upon request to the corresponding author.
